# Serum IL-37 Level Is Associated with Rheumatoid Arthritis and Disease Activity: A Meta-Analysis

**DOI:** 10.1155/2021/6653439

**Published:** 2021-02-05

**Authors:** Shengnan Cao, Haojun Shi, Guodong Sun, Yuanzhen Chen, Guangjian Hou, Dandan Wang, Bin Shi

**Affiliations:** ^1^School of Acupuncture-Tuina, Shandong University of Traditional Chinese Medicine, Jinan 250062, China; ^2^Bone Biomechanics Engineering Laboratory of Shandong Province, Neck-Shoulder and Lumbocrural Pain Hospital of Shandong First Medical University, Jinan 250062, China; ^3^Second Clinical Medical College, Henan University of Chinese Medicine, Henan 450016, China; ^4^Department of Rehabilitation Medicine, The Third Affiliated Hospital of Shandong First Medical University, Jinan 250062, China

## Abstract

Interleukin-37 (IL-37) inhibits the pathogenesis of rheumatoid arthritis (RA) via downregulating proinflammatory cytokines. Accordingly, we performed an analysis to accurately assess the relationship between serum IL-37 cytokine levels and disease activity of RA. Subgroup analysis and sensitivity analysis were applied to explore the sources of heterogeneity. Correlation coefficient (*r*) was utilized to evaluate the relationship between IL-37 and disease activity of RA patients. Ten studies were included into the research. Functional analysis revealed elevated serum IL-37 concentrations in RA patients (SMD = 1.61, *P* < 0.00001). The relationship between serum IL-37 levels and disease activity was statistically significant (C-reactive protein: *r* = 1.47, *P* = 0.0002; erythrocyte sedimentation rate: *r* = 1.55, *P* < 0.00001; rheumatoid factor: *r* = 1.40, *P* = 0.004; tumor necrosis factor⁃*α*: *r* = 1.64, *P* = 0.0003; Disease Activity Score for 28 joints: *r* = 1.63, *P* < 0.00001; tender joint count: *r* = 1.48, *P* < 0.00001; and swollen joint count: *r* = 1.52, *P* = 0.0003), but anti-CCP was not significant (anti-CCP: *r* = 0.98, *P* = 0.72). In summary, these data are suggesting that the elevated serum level of IL-37 in RA is positively correlated with the disease activity of RA, suggesting a role for IL-37in the pathogenesis of RA.

## 1. Introduction

Rheumatoid arthritis (RA) has an estimated prevalence of 1% to 2% worldwide and seriously impacts patients' life quality [1, 2]. Pathological manifestation of RA is chronic inflammation of multiple synovial joints, and progressive inflammation can cause destruction of articular cartilage and bone, eventually leading to irreversible progressive joint deformity and loss of function [3]. In addition, studies showed that interleukin promoted disease development by activating the expression of genes involved in tissue degradation, synovial tissue proliferation, and joint erosion [4]. Targeting Interleukin-17 (IL-17) provides a potential therapy [5]. However, treatment of RA patients with monoclonal antibodies against IL-17 may cause adverse effects [6]. Therefore, the search for new cytokines related to RA and have therapeutic potential is still continuing.

IL-37 is a newly discovered natural immune response inhibitor and exerts anti-inflammatory effects by suppressing proinflammatory cytokines [7]. IL-37 includes five splice variants (IL-37a–e), which have intracellular and extracellular functions same as cytokines [8]. Research demonstrated that IL-37 suppressed certain cells such as macrophages, monocytes, and epithelial cells to secrete proinflammatory cytokines [8]. Abnormal IL-37 expressions in serum have been reported in several inflammation-related diseases, such as RA and ankylosing spondylitis [9, 10]. In in vitro experiments, IL-37 inhibited joint inflammation and significantly reduced the expression of IL-17, IL-1, and IL-6 in Th17 cells. [11]. Studies demonstrate that IL-37 may play a critical role in the pathogenesis of RA. To define the role of IL-37 in the progression of RA, we performed the current meta-analysis.

## 2. Materials and Methods

### 2.1. Literature Search Strategy

This article follows the criteria of the Preferred Reporting Items for Systematic Reviews and Meta-Analyses, with relevant research searched up to November 2020, including the Embase, Web of Science, PubMed, and Chinese National Knowledge Infrastructure (CNKI) databases. The keywords used for search were as follows: “Interleukin-37” or “Interleukin 37” or “IL-37” or “IL 37,” “Rheumatoid Arthritis” or “RA” or “Arthritis, Rheumatoid.” Publication languages were limited to English and Chinese. The search strategy and study selection were independently performed by two researchers on a database search, and the final research choices were agreed upon. Two researchers independently evaluated the same article to determine their eligibility for inclusion and resolved differences through consensus.

### 2.2. Inclusion and Exclusion Criteria

The included researches were based on the following criteria: (1) explored the relationship between serum IL-37 levels and RA; (2) observational studies, such as cross-sectional, case-control, or cohort designs in human; (3) measured the IL-37 level, and/or disease activity in patients and controls must be provided; and (4) the control group must be healthy controls (HCs). Excluded studies were based on the following criteria: (1) do not meet the inclusion criteria; (2) complete data not provided or cannot calculate the required data; (3) cannot obtain the full text or duplicated studies; (4) reviews or comments; and (5) animal research.

### 2.3. Data Extraction

The following information was collected from each study: publication year, country, ethnicity, specimen source, gender and age, case and control numbers, period of RA, and the serum IL-37 level. In addition, the correlation coefficient (*r*) between the IL-37 level and the disease activity was also collected, including erythrocyte sedimentation rate (ESR), C-reactive protein (CRP), anticyclic citrullinated peptide (anti-CCP), rheumatoid factor (RF), Disease Activity Score for 28 joints (DAS28), tender joint count (TJC), swollen joint count (SJC), and TNF-*α*.

### 2.4. Quality Assessment

All studies were assessed using the Newcastle-Ottawa Scale (NOS) assessment scale [12]. The relevant data was independently extracted by two reviewers (Shengnan Cao and Haojun Shi), and disagreement was resolved through discussion and referred to a third reviewer (Bin Shi) if necessary. The scale includes nine items covering three dimensions. A point is awarded for each item that is satisfied by the study. The NOS scores range from 0 to 9, with higher scores indicating higher quality. In this study, score ≥ 6 was defined as high quality.

### 2.5. Statistical Analysis

We used the Review Manager (RevMan 5.3, Cochrane Collaboration, Nordic Cochrane Center, Copenhagen, Denmark) for statistical analyses. The difference between IL-37 in RA and HC was calculated by standardized mean differences (SMDs) and 95% confidence intervals (CIs). When some studies reported results using the median of the first and third quartiles (*M* (*P*_25_, *P*_75_)), an approximation method was used to calculate the mean and standard deviation (*X* ± *S*) [13]: *X* ≈ (*P*_25_ + *M* + *P*_75_)/3 and *S* = (*P*_75_ − *P*_25_)/1.35. Besides, all standard errors of the correlation coefficient (SE) were calculated by the following formula [14]: $\text{SE}=\sqrt{{\left(\left(1-r\right)/\left(n-1\right)\right)}^{2}}$ to combine the *r* of the random-effect model. *Q*-statistic (*P* < 0.05) and *I*^2^ statistics (*I*^2^ > 50%) were used to assess the heterogeneity among studies. In individual studies, we used the Cochrane Collaboration's tool to assess the risk of bias. *P* < 0.05 means statistical significant.

## 3. Results

### 3.1. Included Studies and Quality Assessment

After a comprehensive literature search and verification, the author's research yielded a total of 390 records, of which 47 duplicate records were excluded. Also, 163 nonrelevant studies, 76 nonhuman studies, and 68 conference or comment abstracts were excluded. Finally, 10 studies were eligible for the systematic analysis [15–24] (Figure 1). In total, 731 RA patients were included in this study, of which 529 were females. Data characteristics of the included studies are in Table 1.

### 3.2. Outcomes and Sensitivity Analysis

Through the heterogeneity test, the results showed that the IL-37 level was significantly higher in RA (SMD = 1.61, *P* < 0.00001). Sensitivity analysis showed that the combined SMDs did not change significantly, indicating that our results were stable. The Cochrane Risk of Bias Tool was used to judge the risk of bias for each included study. Though all studies were peer-reviewed and did not address conflicts of interest, most of the included studies did not provide sufficient information to assess overall quality (Figure 2). Small subject numbers can increase heterogeneity and bias; the publication bias was examined using the funnel plot.

### 3.3. Subgroup Analysis

Since heterogeneity existed among included articles, subgroup analysis was performed according to the ethnicity, sample size, and disease period. For ethnicity, the serum IL-37 level of RA patients in Asians (SMD = 1.42, 95%CI = 1.27‐1.58) and African (SMD = 1.75, 95%CI = 1.26‐2.24). According to the sample size stratification, for RA patients, IL-37 levels were identified in both small sample size and large sample size (small: SMD = 4.53, 95%CI = 2.61‐6.46; large: SMD = 1.67, 95%CI = 0.40‐2.95). Furthermore, the significant difference was shown in the disease period (active: SMD = 3.67, 95%CI = 3.23‐4.11; inactive: SMD = 1.86, 95%CI = 1.45‐2.27) (Table 2).

### 3.4. Correlation of IL-37 Level and RA

The relationship between the IL-37 level and disease activity of RA was investigated. The serum IL-37 level was positively correlated with CRP, ESR, RF, and TNF-*α* levels (CRP: *r* = 1.47, *P* = 0.0002; ESR: *r* = 1.55, *P* < 0.00001; RF: *r* = 1.40, *P* = 0.004; TNF-*α*: *r* = 1.64, *P* = 0.0003) (Table 3). In addition to anti-CCP, the DAS28 scores, TJC counts, and SJC counts were also correlated with the IL-37 level (DAS28: *r* = 1.63, *P* < 0.00001; TJC: *r* = 1.48, *P* < 0.00001; SJC: *r* = 1.52, *P* = 0.0003; anti-CCP: *r* = 0.98, *P* = 0.72) (Figure 3).

## 4. Discussion

In this study, we reviewed the literature about the association between serum IL-37 level and RA. The results consistently prove that the IL-37 level in RA was significantly elevated. At the same time, it demonstrated that the IL-37 level was associated with disease activity of RA.

RA is the most commonly diagnosed systemic inflammatory arthritis. Generally, IL-37 is an important anti-inflammatory cytokine involved in inflammation regulation and can inhibit the expression and function of proinflammatory cytokines [25]. Researchers reported that the plasma level of IL-37 was increased in RA [26]. Meanwhile, as demonstrated by authors, IL-37 levels in serum and synovial fluid of RA patients were elevated markedly, whereas they were almost undetectable in healthy controls. Our meta-analysis results showed that when analyzed by ethnic subgroup, in Asian RA patients (mainly Chinese), IL-37 levels were significantly higher than in healthy people. IL-37 was expressed in the thymus, bone marrow, lymph nodes, NK cells, monocytes, and B cells [27]. Studies have shown that IL-37 could be upregulated under the action of inflammatory stimulation and cytokines, such as TLR agonists, IL-1*β*, IL-18, and TNF-*α*. IL-37 may mediate the negative feedback mechanism that inhibits excessive proinflammatory cytokines in RA patients [26]. Accordingly, the increase of anti-inflammatory cytokines IL-37 may be a potential mechanism to reduce the severity of joint inflammation and disease. Series studies have shown that IL-37 may be a potential biomarker for RA diagnosis, disease activity assessment, or curative effect observation [28].

RF form part of the differential diagnosis of arthropathies, and the main index of serological diagnosis of RA. Serological indicators of ESR and CRP are nonspecific inflammatory markers, which have been used to assess systemic inflammatory responses, and have proven diagnostic value for RA. DAS28 is a quantitative index for evaluating RA disease activity [29, 30]. Simultaneously, TJC and SJC are counting tools to detect joint tenderness and swelling. Therefore, we explored the potential relationship between IL-37 levels and related parameters. Results indicated that the CRP, ESR, RF, TNF-*α*, DAS28, TJC, and SJC levels of RA patients were positively correlated with the IL-37 level. Consistent with our findings, researchers reported a positive correlation between the plasma level of IL-37 and both CRP and DAS28 [28]. The TNF-*α* is an important factor leading to the onset of RA, and with the increases of inflammatory response and the proinflammatory cytokine TNF-*α*, IL-37 also increases, which is closely related to disease activities and may play a protective role in the occurrence and development of RA [31, 32]. Anti-CCP antibody is a well-known serological marker [33]. In the diagnosis of early RA, it improves the diagnostic accuracy by measuring the anti-CCP antibody and RF [34]. However, this study used these clinical indicators to explore the relationship between IL-37 levels and RA disease activity and found that the anti-CCP level of RA patients was not correlated with the IL-37 level. This may be caused by the limited number of relevant studies and cases.

However, some limitations should be considered. The meta-analysis results of the included articles were relatively heterogeneous. After subgroup analysis, the source of heterogeneity was not found. This may be due to differences in experimental design and quality, which needs further investigation. At the same time, the insufficient number of related studies and cases is another limit that should also be considered. Finally, RA patients were mainly from Chinese, so our conclusions cannot be extrapolated to other populations.

In all, our meta-analysis provided that the serum IL-37 level is significantly elevated in RA. The serum IL-37 level is positively correlated with disease activity of RA, and further studies are needed to verify our findings.

## Figures and Tables

**Figure 1:** Flow diagram for study selection.

**Figure 2:** Forest plots for SMDs of IL-37 levels with RA and HCs.

**Figure 3:** Forest plot of the C-reactive protein (CRP), erythrocyte sedimentation rate (ESR), anticyclic citrullinated peptide (anti-CCP), rheumatoid factor (RF), Disease Activity Score for 28 joints (DAS28), tender joint count (TJC), swollen joint count (SJC), and tumor necrosis factor-*α* (TNF-*α*).

**Table 1:** Characteristics of eligible studies.

References	Country	Gender		Age		No.		NOS
		Experimental	Control	Experimental	Control	Experimental	Control	
Zhang and Li (2016) [23]	China	M: 17 F: 62	M: 34 F: 66	53.9 ± 9.4	51.7 ± 10.20	79	100	7
Chen and Wang (2014) [19]	China	M: 11 F: 57	M: 4 F: 16	54.41 ± 14.09	53.5 ± 10.55	68	20	7
Song et al. (2018) [16]	China	M: 7 F: 52	M: 17 F: 29	50.4 ± 14.7	44.7 ± 13.70	59	46	7
Yang et al. (2015) [18]	China	M: 83 F: 69	M: 60 F: 40	52.3 ± 15.6	52 ± 14.10	152	100	7
Wu et al. (2019) [21]	China	M: 13 F: 12	NA	48.4 ± 10.16	47.2 ± 9.98	25	25	6
Wan et al. (2016) [20]	China	M: 10 F: 35	M: 6 F: 15	41.3 ± 2.1	41.2 ± 2.30	45	21	6
Xu et al. (2017) [22]	China	M: 12 F: 47	NA	59.86 ± 11.50	NA	59	30	6
Xia et al. (2015) [17]	China	M: 22 F: 128	M: 6 F: 44	51.3 ± 18.6	45.2 ± 20.40	150	50	7
Ragab et al. (2019) [15]	Africa	M: 8 F: 40	M: 7 F: 35	48.67 ± 20.74	44.7 ± 13.70	48	42	6
Akram et al. (2018) [24]	Pakistan	M: 19 F: 27	M: 11 F: 9	54.33 ± 34.07	44.0 ± 12.59	46	20	6

M: male; F: female; No: number; NOS: Newcastle-Ottawa Scale; NA: not available.

**Table 2:** Results of subgroup analysis of included literatures.

Subgroup	*N*	SMD (95% CI)	*Z*	*P*	Heterogeneity		Model
					*I* ^2^ (%)	*P*	
Ethnicity							
Asians	9	1.42 (1.27, 1.58)	18.11	<0.00001	98%	<0.00001	R
African	1	1.75 (1.26, 2.24)	7.01	<0.00001	NA	NA	R
Sample size							
Large	4	1.67 (0.40, 2.95)	2.57	0.01	98%	<0.00001	R
Small	6	1.17 (0.96, 1.37)	11.28	<0.00001	96%	<0.00001	R
Period							
Active	3	3.67 (3.23, 4.11)	16.38	<0.00001	98%	<0.00001	R
Inactive	3	1.86 (1.45, 2.27)	8.93	<0.00001	97%	<0.00001	R
All	10	3.25 (2.21, 4.29)	6.13	<0.00001	98%	<0.00001	R

*N*: number; CI: confidence interval; R: random-effect model; SMD: standard mean difference; NA: not available.

**Table 3:** Correlation between serum IL-37 level and disease activity in RA patients.

Variable	No.	*r*	95% CI	*Z*	*P*	Model
			(LCI, UCI)			
CRP	5	1.47	(1.20, 1.79)	3.73	0.0002	R
ESR	4	1.55	(1.41, 1.71)	9.13	<0.00001	R
Anti-CCP	3	0.98	(0.88, 1.09)	0.36	0.72	R
RF	4	1.40	(1.11, 1.75)	2.89	0.004	R
DAS28	6	1.63	(1.38, 1.93)	5.70	<0.00001	R
TJC	3	1.48	(1.25, 1.77)	4.46	<0.00001	R
SJC	3	1.52	(1.20, 1.93)	3.43	0.0006	R
TNF-*α*	2	1.64	(1.26, 2.13)	3.66	0.0003	R

No: number; CI: confidence interval; R: random-effect model; *r*: correlation coefficient.

## References

[1] Minichiello E., Semerano L., Boissier M. C. (2016). Time trends in the incidence, prevalence, and severity of rheumatoid arthritis: a systematic literature review. *Joint, Bone, Spine*.

[2] Zhou R. P., Wu X. S., Xie Y. Y. (2016). Functions of interleukin-34 and its emerging association with rheumatoid arthritis. *Immunology*.

[3] El-Sayed E. H., Saleh M. H., Al-Shahaly M. H., Toraih E. A., Fathy A. (2018). IL-37 gene variant (rs 3811047): a marker of disease activity in rheumatoid arthritis: a pilot study. *Autoimmunity*.

[4] Sharma J., Bhar S., Devi C. S. (2017). A review on interleukins: the key manipulators in rheumatoid arthritis. *Modern Rheumatology*.

[5] Fleischmann R., Schiff M., van der Heijde D. (2017). Baricitinib, methotrexate, or combination in patients with rheumatoid arthritis and no or limited prior disease-modifying antirheumatic drug treatment. *Arthritis & Rheumatology*.

[6] Wei M., Duan D. (2016). Efficacy and safety of monoclonal antibodies targeting interleukin-17 pathway for inflammatory arthritis: a meta-analysis of randomized controlled clinical trials. *Drug Design, Development and Therapy*.

[7] Xu W. D., Zhao Y., Liu Y. (2015). Insights into IL-37, the role in autoimmune diseases. *Autoimmunity Reviews*.

[8] Boraschi D., Lucchesi D., Hainzl S. (2011). IL-37: a new anti-inflammatory cytokine of the IL-1 family. *European Cytokine Network*.

[9] Chen B., Huang K., Ye L. (2015). Interleukin-37 is increased in ankylosing spondylitis patients and associated with disease activity. *Journal of Translational Medicine*.

[10] Ye L., Ji L., Wen Z. (2014). IL-37 inhibits the production of inflammatory cytokines in peripheral blood mononuclear cells of patients with systemic lupus erythematosus: its correlation with disease activity. *Journal of Translational Medicine*.

[11] Wang X., Xu K., Chen S., Li Y., Li M. (2018). Role of interleukin-37 in inflammatory and autoimmune diseases. *Iranian journal of Immunology*.

[12] Stang A. (2010). Critical evaluation of the Newcastle-Ottawa scale for the assessment of the quality of nonrandomized studies in meta-analyses. *European Journal of Epidemiology*.

[13] Wan X., Wang W., Liu J., Tong T. (2014). Estimating the sample mean and standard deviation from the sample size, median, range and/or interquartile range. *BMC Medical Research Methodology*.

[14] Cai G., Wang L., Fan D. (2015). Vitamin D in ankylosing spondylitis: review and meta-analysis. *Clinica Chimica Acta*.

[15] Ragab D., Mobasher S., Shabaan E. (2019). Elevated levels of IL-37 correlate with T cell activation status in rheumatoid arthritis patients. *Cytokine*.

[16] Song L., Wang Y., Sui Y. (2018). High interleukin-37 (IL-37) expression and increased mucin-domain containing-3 (TIM-3) on peripheral T cells in patients with rheumatoid arthritis. *Medical Science Monitor*.

[17] Xia L., Shen H., Lu J. (2015). Elevated serum and synovial fluid levels of interleukin-37 in patients with rheumatoid arthritis: attenuated the production of inflammatory cytokines. *Cytokine*.

[18] Yang L., Zhang J., Tao J., Lu T. (2015). Elevated serum levels of interleukin-37 are associated with inflammatory cytokines and disease activity in rheumatoid arthritis. *APMIS*.

[19] Chen H. X., Wang X. F. (2014). Role of IL-37 in the pathogenesis of rheumatoid arthritis. *Journal of China Medical University*.

[20] Wan L. L., Wang X. D., Ci Z. C. (2016). Expression of TLR4 in peripheral blood of patients with 274 rheumatoid arthritis and its correlation with IL-37 level. *World Journal of Complex Medicine*.

[21] Wu H. M., He S. Q., Zhou D., Huang Z., Hu G. T., Zhang F. (2019). Clinical significance of serum IL-37 detection in patients with rheumatoid arthritis. *Journal of Clinical Transfusion and Laboratory Medicine*.

[22] Xu W. M., Xu J., Wan Y. (2017). Clinical significance of serum IL-37 detection in patients with rheumatoid arthritis. *Journal of Clinical Transfusion and Laboratory Medicine*.

[23] Zhang J. F., Li Y. L. (2016). Clinical significance of detection of serum IL-37 and IL-10 levels in patients with rheumatoid arthritis. *Medical Journal of Chinese People’s Health*.

[24] Akram N., Jamal A., Ullah S. (2018). Expression level of serum interleukin-37 in rheumatoid arthritis patients and its correlation with disease activity score advancements in. *Life Sciences*.

[25] Nold M. F., Nold-Petry C. A., Zepp J. A., Palmer B. E., Bufler P., Dinarello C. A. (2010). IL-37 is a fundamental inhibitor of innate immunity. *Nature Immunology*.

[26] Xia T., Zheng X.-f., Qian B.-h. (2015). Plasma interleukin-37 is elevated in patients with rheumatoid arthritis: its correlation with disease activity and Th1/Th2/Th17-related cytokines. *Disease Markers*.

[27] Jia H., Liu J., Han B. (2018). Reviews of interleukin-37: functions, receptors, and roles in diseases. *BioMed Research International*.

[28] Zhao P. W., Jiang W. G., Wang L., Jiang Z. Y., Shan Y. X., Jiang Y. F. (2014). Plasma levels of IL-37 and correlation with TNF-*α*, IL-17A, and disease activity during DMARD treatment of rheumatoid arthritis. *PLoS One*.

[29] Zhang X., Yuan Y., Pan Z. (2019). Elevated circulating IL-17 level is associated with inflammatory arthritis and disease activity: a meta-analysis. *Clinica Chimica Acta*.

[30] do Prado A. D., Bisi M. C., Piovesan D. M. (2016). Ultrasound power Doppler synovitis is associated with plasma IL-6 in established rheumatoid arthritis. *Cytokine*.

[31] Atzeni F., Talotta R., Masala I. F., Bongiovanni S., Boccassini L., Sarzi-Puttini P. (2017). Biomarkers in rheumatoid arthritis. *The Israel Medical Association Journal*.

[32] Wells A. F., Curtis J. R., Betts K. A., Douglas K., Du E. X., Ganguli A. (2017). Systematic literature review and meta-analysis of tumor necrosis factor-alpha experienced rheumatoid arthritis. *Clinical Therapeutics*.

[33] Vos I., Van Mol C., Trouw L. A. (2017). Anti-citrullinated protein antibodies in the diagnosis of rheumatoid arthritis (RA): diagnostic performance of automated anti-CCP-2 and anti-CCP-3 antibodies assays. *Clinical Rheumatology*.

[34] Ingegnoli F., Castelli R., Gualtierotti R. (2013). Rheumatoid factors: clinical applications. *Disease Markers*.

